The article "Exosomal SNHG16 secreted by CSCs promotes glioma development via TLR7" was retracted in 2022. Reasons: unreliable results or conclusions; lack of ethics approval or compliance; concerns about the data; concerns about the results or conclusions.

# Exosomal SNHG16 secreted by CSCs promotes glioma development via TLR7

**DOI:** 10.1186/s13287-021-02393-8

**Published:** 2021-06-16

**Authors:** Ruijie Zhang, Peng Li, Heli Lv, Nana Li, Suliang Ren, Wentao Xu

**Affiliations:** 1 Department of Neurology, Heze Hospital of Traditional Chinese Medicine, Heze, 274000 Shandong China; 2 Department of Neurosurgery, Heze Hospital of Traditional Chinese Medicine, 1036, Danyang Road, Heze, 274000 Shandong China; 3 Department of Non-treatment, Wenshang County Hospital of Traditional Chinese Medicine, Jining, 272501 Shandong China

**Keywords:** Glioma, Exosome, CSC, SNHG16, TLR7

## Abstract

**Background:**

Glioma is one of the most common central nervous system malignant tumors, accounting for 45~60% of adult intracranial tumors. However, the clinical treatment of glioma is limited. It is of great significance to seek new therapeutic methods for glioma via gene therapy.

**Methods:**

Long non-coding RNA (lncRNA) SNHG16 expression level was measured by microarray and qRT-PCR assay; ISH was used to identify the location of SNHG16. Cancer stem cells (CSCs) were separated from glioma tissues and identified using immunofluorescence. Exosomes were isolated from CSCs and cancer cells and identified by TEM and western blot. MTT, wound healing, transwell, and colony formation assay were performed to explore the role of SNHG16 or si-SNHG16 from CSCs on progression of glioma cells. RIP was used to verify the interaction between SNHG16 and TLR7. The experiment of Xenograft used for exploring the function of SNHG16/ TLR7/MyD88/NFκB/c-Myc on growth on glioma in vivo.

**Results:**

Microarray assay showed long non-coding RNA (lncRNA) SNHG16 was upregulated in glioma. Followed qRT-PCR also showed an increase of SNHG16 in glioma tissues; high expression of SNHG16 indicated a poor prognosis in glioma patients. Interestingly, SNHG16 was packaged into exosomes and derived from CSCs. Functional analysis showed exo-SNHG16 secreted by CSCs promoted the progression of glioma cell lines SHG44 and U251. Furthermore, SNHG16 interacted with TLR7 and activated NFκB/c-Myc signaling in glioma cells. And the silencing of TLR7 inhibited the progression of SHG44 and U251 cells by exo-SNHG16 from CSCs. In vivo tumorigenesis experiments showed that exo-SNHG16 induced glioma progression by activating TLR7/MyD88/NFκB/c-Myc signaling.

**Conclusion:**

Our study suggested CSC-derived exo-SNHG16 promoted cancer progression by activating TLR7/MyD88/NFκB/c-Myc signaling pathway.

**Supplementary Information:**

The online version contains supplementary material available at 10.1186/s13287-021-02393-8.

## Background

Glioma, a common malignant tumor in CNS, accounting for 45~60% of adult intracranial tumors [1]. Since malignant glioma growth is invasive, glioma is prone to relapse and migration, which significantly increases clinical treatment difficulty [2]. Surgical resection and radiotherapy are the main methods for glioma treatment, but can only treat the symptoms rather than the root cause. Postoperative patients often have recurrence or metastasis, which dramatically reduces the postoperative survival rate [3]. In recent years, gene therapy for glioma has become a hot research field [4]. Thus, it is of great significance to find the treatment of glioma from the perspective of molecules.

Long non-coding RNA (lncRNA) was considered as a transcription noise without biological function. Still, now it has been found that lncRNA not only participates in critical biological processes, such as epigenetic regulation, transcription, and post-transcriptional regulation [5, 6] but is also closely related to a variety of tumorigenesis and development [7]. Recent studies have found that lncRNA also contributes to the development of glioma [8] and closely relates to patients' prognosis [9, 10]. MEG3(maternally expressed 3) can interact with cAMP, p53, MDM2, and GDF15 to regulate cell proliferation [11]. In glioma cell lines, overexpression of MEG3 inhibited cell proliferation and promoted apoptosis. Further studies have found that it may inhibit tumorigenesis and development by selectively activating downstream gene transcription after activating p53 [12]. Therefore, MEG3 may play the role of the tumor suppressor gene in glioma. It has been reported that lncRNA SNHG16 acted as an oncogene to promote tumor development in breast cancer, gastric cancer and other cancers [13, 14]. However, the roles and mechanism of SNHG16 in glioma have not been thoroughly identified.

Exosomes are vesicles with a size of 30~100 nm that originate from endosomes [15]. Exosomes are important mediators of intercellular transport and communication, which participate in various physiological and pathological processes of cells [16]. Cancer stem cells (CSCs) are a special type of tumor cells with differentiation and self-renewal potential and exist in various tumor tissues [17]. Some studies have pointed out that the main reason for the failure of most clinical cancer treatment is CSC’s existence and its high differentiation ability [18]. In fact, there is a dynamic equilibrium state between CSCs and non-CSCs [19]. In specific microenvironments, non-CSCs can regain the stem phenotype through dedifferentiation or reprogramming. CSCs and non-CSCs maintain their dynamic balance by communicating between cells. In particular, exosomes are essential carriers for cell communication between CSCs and non-CSCs in tumor process [20]. It has been reported that six lncRNAs were identified in exosomes of HeLa and McF-7 cells [21]. However, exosomal lncRNA’s role in the transformation of non-CSCs and CSCs of glioma has been rarely investigated.

In this study, we explored the function of exosomal SNHG16 in the transformation of non-CSCs and CSCs in glioma and further investigated the underlying mechanisms.

## Methods

### Tissue specimen

The surgical specimens (normal para-carcinoma tissues and cancerous tissues) of 30 giloma patients from were collected and stored in liquid nitrogen. And glioma tissues were collected from grade I to grade IV glioma patients; the grade tissues were from 6 patients. All the patients signed informed consent, and our experiment was permitted by the Ethics Review Committee of Heze Hospital of Traditional Chinese Medicine and the patients signed informed consent.

### CSCs and exosome isolation and identification

CSCs and cancer cells (CCs) were isolated from cancer and para-carcinoma tissues of glioma patients as previous described [22], which identified with CD105 and Nestin. And CSCs were cultured in DMEM-F12 (Gibco, USA) with 10 ng/ml bFGF (Wolcavi, China), 20 ng/ml EGF (Sigma, USA), 5 μg/ml insulin (Sigma, USA), and 0.4% BSA (Sigma, USA). Exosomes in culture medium were isolated using several centrifugations. Transmission electron microscopy (TEM) was used to identify exosomes structures [22]. CSC-derived exosomes were analyzed using exosome marker protein CD63 (ab134045, Abcam), Tsg101 (ab125011, Abcam), and ALIX (ab275377, Abcam) via Western blot.

### Cell culture and treatment

We purchased glioma cell lines (SHG44 and U251) from ATCC cell center of The United States, which are two commonly used cell lines in glioma. The cells were cultured with complete medium including 1640 medium with 10% fetal bovine serum and 1% dual-antibody solution in an incubator at 37 °C and 5% CO_2_. Two micrograms of plasmid or small interfering RNA (si-RNA) was transfected into cells, which was mediated by LipofectamineTM 2000 (Invitrogen, Carlsbad, CA, USA). And plasmid or miRNA or small interfering RNA (si-RNA) were constructed and purchased from by Ribobio company (Guangzhou, China); 5 μg/ml exosomes were added into the medium of cells every 24 h.

### qRT-PCR

We used trizol method to extract RNA in tissues and cells, and RNA concentration and purity were determined using NanoDrop 2000 (Thermo Scientific, USA). RNA is used as transcription template to reverse transcribe into cDNA. Then, SYBR Premix Ex TaqII was selected for RT PCR reaction. The expression value of the normal group was set as 1, and the relative expression of the experimental group was expressed as 2-△△CT. GAPDH was used as internal control. Primer list is as follows: SNHG16 (F: CCTCTAGTAGCCACGGTGTG, R: GGCTGTGCTGATCCCATCTG), TLR7 (F: TAGGATCACTCCATGCCATCAA, R: CAGTGTCCACATTGGAAACACC), GAPDH (F: AGATCATCAGCAATGCCTCCTG, R: ATGGCATGGACTGTGGTCATG).

### Western blot

The tissue or treated cells were lysed firstly. After centrifugation, the supernatant was separated and placed in a 0.5-mL centrifuge tube. BCA method was used to determine the concentration of each sample, and protein loading treatment and quantitative protein samples were used. The samples were electrophoretic with polyacrylamide gel and then transferred to PVDF membrane. The PVDF membrane carrying protein was sealed with 1%BSA for 2 h and incubated with primary antibody at 4 °C overnight. The second antibody was incubated the next day, and the amount of protein samples on the PVDF membrane was detected by chemical radiography. The antibodies are as follows: TLR7 (17232-1-AP, Proteintech), p65 (10745-1-AP, Proteintech), p50 (14220-1-AP, Proteintech), Histone H1 (15446-1-AP, Proteintech), cMyc (10828-1-AP, Proteintech), and GAPDH (60004-1-Ig, Proteintech).

### MTT assay

MTT assay was used to determine the proliferative ability of SHG44 and U251 cells. One hundred microliters (1 × 10^4^ cells) was inoculated in 96-well plates and cultured at 37 °C with 5% CO_2_ for 24 h. At 24 h after transfection, 50 μL MTT solution (5 mg/mL) was added to each well, and the supernatant was discarded after incubation for 4 h at 37 °C. The reduction reaction was terminated by adding 150 μL dimethyl sulfoxide (DMSO) to each well. The 96-well plate was continuously shaken for 30 min, the optical density value of each well at 570 nm wavelength was determined by ELISA, and the average value of each group was taken.

### Immunohistochemistry (IHC) assay

Paraffin sections of carcinoma were dewaxed to water in xylene and descending series of ethanol. We penetrated sections using 0.5% Triton X-100. After 3 times of washing, we blocked sections with 50% goat serum. Then, the sections were incubated with Ki67 antibody (ab15580, Abcam) overnight. On the second day, tumor sections were incubated with secondary antibody for 1 h, and then stained nuclei using DAPI for 5 min. Then, IHC staining positive region were detected by microscope under light scope.

### Cell migration assay

SHG44 and U251 cells were cultured in a 6-well culture plate, and after 24 h of growth at a density, they should achieve a monolayer fusion of about 70–80%. Gently and slowly scrape a single layer with the tip of a new 200-μl pipette through the center of the hole. After scraping, wash the hole gently with medium twice to remove the isolated cells. The cells were cultured in a fresh serum-free medium. Cell migration was recorded at 0 h and 24 h after culture.

### Cell invasion assay

The matrix glue and basic medium 1640 were fully mixed according to 1:3. A mixture of 50 μL matrix glue and basal medium 1640 was added to the bottom of the chamber. The culture plates with small chambers were placed in a 5% CO_2_ incubator for 30 min. Single-cell suspension was prepared, and the cell concentration was adjusted to l × 10^5^/mL. In the 24-well plate, a small chamber with and without coated matrix glue was set, and a complete medium containing 10% serum was added. Cell suspension of 200 μL was slowly added into a small chamber and cultured at 37 °C and 5% CO_2_ for 24 h. The cells in the small chamber were removed with a wet cotton swab and fixed immediately with formaldehyde for 5 min. After that, the small chamber was taken out and dried. Crystal violet was used for dyeing for 20 min. Then, the chamber was rinsed with water and dried. The number of transmembrane cells was observed and counted under the microscope.

### EMSA

Electrophoretic MobilityShift Assay kit (PIERCE, USA) was used to determine NFκB activity. According to the reaction system in the procedures, we first prepared NFκB probe complex and purified it. NFκB expression levels were then measured using a nondenatured polyacrylamide gel.

### RNA-binding protein immunoprecipitation (RIP)

We performed an RIP assay to determine the binding between SNHG16 and TLR7/TLR8 using Magna RIP™ RNA-Binding Protein Immunoprecipitation Kit (Millipore) as in the previous study [23]. Briefly, SHG44 and U251 cells were transfected with biotinylated TLR7 or TLR8, and the expression of SNHG16 was detected using qRT-PCR.

### In situ hybrization (ISH)

ISH assay was used to identify the location of SNHG16 in glioma tissues, which was performed as in the previous study [24]. Briefly, SNHG16 probe was constructed by Invitrogen, glioma tissues were incubated with probe hybridization solution, and the images were observed under the microscope.

### Animal experiment

SHG44 and U251 cells of each group were prepared for inoculation for subculture for 15 generations, and the concentration was adjusted to 5 × 10^7^/0.1 ml/site and then divided into different packs. The cell suspension is blown away. Eighteen BALB/C female nude mice 4–5 weeks, with weight around 20 g, were selected and grouped and numbered. Each nude mouse was weighed. The right armpit was disinfected with 75% alcohol, and 0.1 ml cell suspension was injected. And 200 μg exosomes were administered into mice via tail vein injection once every 3 days for 2 weeks. Then, the mice were observed daily. After 4 weeks, the nude mice were collected and killed by excessive carbon dioxide, the tumors were removed, and the tumors were photographed, weighed, and recorded after all the surrounding connective tissues were removed. The animal study was reviewed and approved by the Heze Hospital of Traditional Chinese Medicine.

### Statistical analysis

Data were shown as mean ± SD. Student’s t test or one-way ANOVA was used to compare the groups. *P* < 0.05 was considered significance. All experiments were repeated three times.

## Results

### High level of lncRNA SNHG16 indicated a poor prognosis in glioma patients

We first performed microassay analysis, and the data showed the differentially expressed lncRNAs in normal and cancer tissues (Fig. 1A). Then, qRT-PCR analysis used to confirm the expression of SNHG16 in glioma, which showed that SNHG16 was upregulated in glioma tissues (Fig. 1B). Kaplan-Meier curves used to show the effect of SNHG16 on glioma patients’ survival, which indicated that high expression of SNHG16 inhibited patients’ 7-year survival rate (Fig. 1C). Furthermore, glioma tissues were collected from different grades patients (grade I to grade IV, *n* = 6) and found that the expression level of SNHG16 was positively correlated with the tumor grade (Fig. 1D). Then, ISH assay was used to identify the location of SNHG16 in glioma tissues, which showed that SNHG16 was present in both cytoplasm and nucleus of glioma cells (Fig. 1E).

**Fig. 1:** The expression of lncRNA SNHG16 in glioma tissues. **A** LncRNA expression profiles in normal tissues and cancer tissues of glioma. **B** qRT-PCR analysis of lncRNA SNHG16 in glioma cancerous tissues and normal tissues determined by qRT-PCR (*p < 0.05), *n* = 15. **C** The 7-years’ survival rate of glioma patients with low or high expression of SNHG16 (*p < 0.05), *n* = 7. **D** The expression of SNHG16 in glioma tissues from patients with tumor grade I to grade IV (*n* = 6) was measured by qRT-PCR (*p < 0.05 vs grade I). **E** ISH showed the location of SNHG16 in glioma tissues

### SNHG16 was packaged into exosomes and derived from CSCs

To determine the origin of SNHG16 in glioma, we isolated CSCs from glioma cancer tissue; immunofluorescence assay was performed to identify the markers CD105 and Nestin for CSCs (Fig. 2A). Then, we performed qRT-PCR analysis to determine SNHG16 expression cancer cells (CCs) and CSCs in six glioma patients (case 1#-case 6#). The expression of SNHG16 was increasing in CSCs than that in CCs (Fig. 2B). Furthermore, exosomes in CCs and CSCs were isolated. TEM data showed the morphology of exosomes (Fig. 2C), which indicated there is no difference in morphology of exosomes of cancer cells or CSCs. Then, exosome markers were detected in exosomes from CCs and CSCs, and cell pellet acted as a negative control (Fig. 2D). Interestingly, SNHG16 level was higher in CSC exosomes compared with CC exosomes (Fig. 2E), which indicated that SNHG16 could be packaged into exosomes and derived from CSCs.

**Fig. 2:** CSCs secreted exosomal SNHG16 in glioma. **A** Immunofluorescence staining for CD105 and Nestin expression of CSCs. DAPI indicates nucleus. Scale bar = 20 μm. **B** qRT-PCR analyzed the expression of SNHG16 in cancer cells and CSCs in six glioma patients (case 1#-case 6#). *n* = 6, *p < 0.05. **C** TEM of exosomes isolated from cancer cells and CSCs. Scale bar = 200 nm. **D** Western blot for CD63, Tsg101, and Alix in exosomes. **E** qRT-PCR determined the expression of SNHG16 in isolated exosomes in six glioma patients (case 1#-case 6#). *n* = 6, *p < 0.05

### Exosomal-SNHG16 accelerated cancer progression of glioma cells

To evaluate the role of exosomal-SNHG16 (exo-SNHG16) in glioma development, SHG44 and U251 cells were incubated with exosomes isolated from CSCs transfected SNHG16 or si-SNHG16 or its NC. We first detected SNHG16 expression in isolated exosomes and found SNHG16 transfection induced SNHG16 expression, while si-SNHG16 transfection reduced SNHG16 expression (Fig. 3A, Supplementary figure 1A). Then, we discovered that SNHG16 expression was significantly upregulated in SHG44 and U251 cells upon incubation with exosomes from CSCs with SNHG16 overexpression but not with CSCs with si-SNHG16 (Fig. 3B, Supplementary figure 1B). Functionally, we performed MTT assay to estimate cell viability. It showed that CSCs transfected with SNHG16 increased cell viability, while knockdown of SNHG16 decreased cell viability in SHG44 and U251 cells (Fig. 3C). Furthermore, wound healing assay suggested that CSCs transfected with SNHG16 promoted cell migration in SHG44 and U251 cells (Fig. 3D), but CSCs transfected with si-SNHG16 showed an opposite effect (Fig. 3E). Transwell assay showed that CSCs transfected with SNHG16 induced cell invasion in SHG44 and U251 cells (Fig. 3F), but CSCs transfected with SI-SNHG16 showed an opposite effect (Fig. 3G). In addition, overexpression of SNHG16 promoted proliferation of SHG44 and U251 cells (Fig. 3H), while silencing SNHG16 inhibited proliferative ability (Fig. 3I). Together, exo-SNHG16 secreted by CSCs promoted tumor progression in glioma cells.

**Fig. 3:** Exosomal SNHG16 from CSCs promoted proliferation, migration and invasion. SHG44 and U251 cells were incubated with exosomes isolated from CSCs transfected SNHG16 or si-SNHG16 or its NC. **A** qRT-PCR analyzed the expression of SNHG16 in isolated exosomes. **B** The expression of SNHG16 in SHG44 and U251cells was determined. *n* = 6, *p < 0.05 vs CSC-NC or CSC-si-NC. **C** MTT was used to test viability of SHG44 and U251. *n* = 10, *p < 0.05 vs CSC-NC or CSC-si-NC. **D**, **E** Would healing assay to detect migration ability. Scale bar = 500 μm. *n* = 4, *p < 0.05 vs CSC-NC or CSC-si-NC. **F**, **G** Transwell assay to detect invasion ability. Scale bar = 200 μm. *n* = 4, *p < 0.05 vs CSC-NC or CSC-si-NC. **H**, **I** Colony formation assay to detect cell proliferation. Scale bar = 10 mm. *n* = 6, *p < 0.05 vs CSC-NC or CSC-si-NC

### SNHG16 interacted with TLR7 and activated NFκB/c-Myc signaling

Considering that TLR7 can be activated by single-stranded oligonucleotides and is involved in various disease progression [25], we speculated TLR7 might participate in the process of SNHG16 regulating glioma. To test our hypothesis, SHG44 and U251 cells were incubated with exosomes isolated from CSCs transfected si-SNHG16 or its NC. TLR7 expression was significantly downregulated upon incubation with exosomes from CSCs with si-SNHG16 (Fig. 4A). As well, western blot also showed that si-SNHG16 inhibited the protein expression of TLR7 in SHG44 and U251 cells (Fig. 4B). We performed RNA pull-down assay to explore the relationship between SNHG16 and TLR17 further. Data showed that TLR7 were pulled down with the sense strand of SNHG16 bot not the empty beads in SHG44 and U251 cells (Fig. 4C). And there was a significant enrichment of SNHG16 bound to TLR7 comparing with the IgG in SHG44 and U251 cells (Fig. 4D). Considering the similarity of TLR7 and TLR8, we further analyzed whether SNHG16 could bind with TLR8. The enrichment assay showed a higher SNHG16 expression in TLR8 group than that in IgG group, which was lower than that in TLR7 group (Fig. 4D). Moreover, we found that TLR7 and SNHG16 were co-locations in the cytoplasm (Fig. 4E).

**Fig. 4:** SNHG16 activated TLR7- NFκB-c-Myc signaling pathway. SHG44 and U251 cells were incubated with exosomes isolated from CSCs transfected si-SNHG16/si-NC. **A** qRT-PCR analyzed the expression of TLR7 in SHG44 and U251 cells. *n* = 6, *p < 0.05. **B** Western blot for TLR7 expression in SHG44 and U251 cells. *n* = 4, *p < 0.05. **C** Western-blotting validation of TLR7 in SNHG16 pulldown protein extractions. **D** RNA-immunoprecipitation experiments were performed using TLR7, TLR8 and IgG antibodies to immunoprecipitate SNHG16 in SHG44 and U251 cells. **E** FISH assay was used to detected the subcellular location of SNHG16 and TLR7 in U251 cells, the nucleus was stained using DAPI. Scale bar = 25 μm. **F** NFκB activities was examined by EMSA. *n* = 4, *p < 0.05. **G** Western blotting showing nuclear p65, p50, Histone H1 and c-Myc levels in SHG44 and U251 cells. *n* = 4, *p < 0.05

It has been reported that TLRs activated NFκB and c-Myc through MyD88 in various cancers [26, 27]. Thus, we wonder about the role of SNHG16 on NFκB/c-Myc signaling. SHG44 and U251 cells were incubated with exosomes isolated from CSCs transfected SNHG16, si-SNHG16 or its NC. EMSA data showed that overexpression of SNHG16 promoted NFκB activity, while si-SNHG16 inhibited NFκB activity in SHG44 and U251 cells (Fig. 4F). As well, SNHG16 increased the protein expression of p65, p50 and c-Myc, whereas loss of SNHG16 decreased their expression (Fig. 4G). Taken together, SNHG16 secreted by CSCs could bound with TLR7, and activated NFκB/c-Myc signaling pathway in glioma cells.

### Silencing of TLR7 blocked the promoting effect of exo-SNHG16 on glioma progression

To clarify whether SNHG16 promoted glioma progression by regulating TLR7 in glioma cells, SHG44 and U251 cells were transfected with TLR7 or si-TLR7 and incubated with exosomes from CSCs transfected with SNHG16 or si-SNHG16, respectively. qRT-PCR assay showed that si-TLR7 decreased TLR7 expression, while TLR7 transfection increased TLR7 expression (Fig. 5A, B). Followed functional experiments showed that silencing of TLR7 reduced cell viability, migration, invasion, and proliferation in SHG44 and U251 (Fig. 5C, E, G, I), while overexpression of TLR7 showed the opposite function (Fig. 5D, F, H, J). Thus, silencing of TLR7 inhibited the progression of SHG44 and U251 cells by exo-SNHG16 from CSCs.

**Fig. 5:** SNHG16 maintained cancer stem-like cell dynamic via activating TLR7. SHG44 and U251 cells were transfected with TLR7 or si-TLR7 and incubated with exosomes from CSCs transfected with SNHG16 or si-SNHG16, respectively. **A**, **B** qRT-PCR for mRNA expression of TLR7 in SHG44 and U251 cells. *n* = 4, *p < 0.05. **C**, **D** MTT for cell viability in SHG44 and U251 cells. *n* = 10, *p < 0.05. **E**, **F** Would healing assay for cell migration in SHG44 and U251 cells. Scale bar = 500 μm. *n* = 4, *p < 0.05. **G**, **H** Transwell assay for cell invasion in SHG44 and U251 cells. Scale bar = 200 μm. *n* = 4, *p < 0.05. **I**, **J** Colony formation assay for cell proliferation in SHG44 and U251 cells. Scale bar = 10 mm. *n* = 6, *p < 0.05

### The activation of TLR7/MyD88/NFκB/c-Myc contributed to SNHG16-mediated cancer stem cell transition

The role and underlying mechanism of CSC-derived exo-SNHG16 in glioma development were further evaluated in vivo. SHG44 and U251 cells that stable expressed si-TLR7 were injected into nude mice (*n* = 10), and a dosage of 200 μg exosomes was administered into mice via tail vein injection once every 3 days for 2 weeks. Tumors grew faster and bigger in the mice with CSCs-SNHG16, while si-TLR7 inhibited the growth rate and volume of tumors (Fig. 6A, B). The tumors were isolated at 28 days after injection, CSCs-SNHG16 significantly increased tumors weight, and si-TLR7 removed the promoting role of CSCs-SNHG16 (Fig. 6C, D). In addition, immunohistochemical assay showed CSCs-SNHG16 induced the expression of Ki67, while si-TLR7 reduced Ki67 level (Fig. 6E). Then, EMSA and western blot results indicated that incubation with exosomes from CSCs transfected with SNHG16 increased NFκB activity and c-Myc expression in glioma tumors (Fig. 6F, G).

**Fig. 6:** TLR7 activation was responsible for SNHG16-mediated cancer stem cell transition in vivo. SHG44 and U251 cells that stable expressed si-TLR7 were incubated with exosomes from CSCs transfected with SNHG16 or NC, and then SHG44 and U251 cells were injected into nude mice (*n* = 10). **A**, **B** Growth of tumor xenografts in nude mice. *n* = 10, *p < 0.05. **C**, **D** Representative tumors excised from xenografts in nude mice and tumor weight. *n* = 4, *p < 0.05. **E** Immunofluorescence staining for Ki67 to test proliferation viability. Scale bar = 50 μm. *n* = 4, *p < 0.05. **F** NFκB activities was examined by EMSA. *n* = 4, *p < 0.05. **G** Western blotting for c-Myc expression. *n* = 4, *p < 0.05

MyD88 is the upstream molecule, and then we focused on MyD88 function. SHG44 and U251 cells that stable expressed si-MyD88 were injected into nude mice, and exosomes were administered into mice via tail vein injection once every 3 days for 2 weeks. As expected, si-MyD88 inhibited growth rate, volume, and weight of glioma (Fig. 7A–D). In addition, si-MyD88 inhibited the proliferation of glioma cells (Fig. 7E). Furthermore, deficiency of MyD88 decreased NFκB activity and c-Myc expression in glioma tumors (Fig. 7F, G). Together, these results indicated that exo-SNHG16 induces glioma progression by activating TLR7/MyD88/NFκB/c-Myc signaling pathway.

**Fig. 7:** MyD88 contributed to SNHG16-mediated cancer stem cell transition in vivo. SHG44 and U251 cells that stable expressed si-MyD88 were incubated with exosomes from CSCs transfected with SNHG16 or NC, and then SHG44 and U251 cells were injected into nude mice (*n* = 10). **A**, **B** Tumor growth curve in nude mice. *n* = 10, *p < 0.05. **C**, **D** Representative tumors and tumor weight. *n* = 4, *p < 0.05. **E** Immunofluorescence staining for Ki67 expression. Scale bar = 50 μm. *n* = 4, *p < 0.05. **F** EMSA for NFκB activities. *n* = 4, *p < 0.05. **G** Western blotting for c-Myc expression. *n* = 4, *p < 0.05

## Discussion

Gliomas originate in the neuroepithelium and affect the function of brain tissues, including sensation, movement, cognition, and language [1]. Glioma seriously affects the quality of life of patients and brings a significant burden to the society. Duo to the limitation of clinical treatment, it is of considerable significance to actively seek new methods for glioma treatment. LncRNA, as an essential gene regulatory molecule, s inextricably linked to glioma [28]. Therefore, more and more attention has been paid to the expression and role of lncRNA in glioma.

LncRNA SNHG16 is the first lncRNA found in neuroblastoma. The expression of SNHG16 is tissue-specific, which makes it a diagnostic marker. Studies have reported that SNHG16 plays a crucial effect in many cell progressions [29]. Lu et al. [30] found SNHG16 was increased in glioma tissues and cells, and silencing SNHG16 inhibits the tissue activity. Consistent with the above findings, our study showed that lncRNA SNHG16 was induced in cancer tissues, and the SNHG16 level was positively related with the clinical grade of glioma, which indicated a poor prognosis in glioma patients.

Studies have shown that the presence of CSCs is the leading cause of tumor growth, development, and recurrence [31]. Non-cancer stem cells (NCSCs) and CSCs can transform each other, which maintains the dynamic balance of CSCs [32]. In particular, exosomes mediate communication between NCSCs and CSCs, thus keeping the dynamic balance of CSCs [33]. Here, SNHG16 had a higher level in exosomes from CSCs than that in cancer cells, which indicated that SNHG16 was packaged into exosomes and derived from CSCs. Functional analysis showed exo-SNHG16 secreted by CSCs promoted progression of glioma cell lines SHG44 and U251.

TLRs is a pattern recognition receptor, which was initially found to be mainly expressed in various immune cells and involved in the immune response [34]. Moreover, TLRs is related to tumor development, including gastric cancer, colorectal cancer, ovarian cancer, and glioma [35, 36]. NFκB is a critical molecule that connects chronic inflammation with tumors, and the activation of NFκB can directly stimulate the growth and development of tumors [37]. Specially, TLRs can promote the expression and activation of NFκB, thus improving the aggregation of immune cells and the production of anti-apoptotic factors, ultimately inducing angiogenesis and promoting tumor growth and progression by inhibiting apoptosis and cytotoxicity [38, 39]. In our study, we found that lncRNA SNHG16 interacted with TLR7 and activated NFκB/c-Myc signaling in glioma cells. TLR7 and TLR8 are highly similar; we further examine the binding between SNHG16 and TLR8; the enrichment assay also showed a increasing level of SNHG16 in TLR8, which is lower than that in TLR7 group. And this data indicated SNHG16 mainly bond with TLR7. Further functional experiments showed that silencing of TLR7 inhibited the progression of SHG44 and U251 cells by exo-SNHG16 from CSCs. In vivo tumorigenesis experiments showed that exo-SNHG16 induced glioma progression by activating TLR7/MyD88/NFκB/c-Myc signaling pathway (Fig. 8).

**Fig. 8:** Hypothesis diagram illustrates function and mechanism of exosomal SNHG16 from CSCs in glioma progress

Though the present study showed that SNHG16 derived from CSCs mediates the development of glioma both in vitro and in vivo, there were still some limitations. The progression of glioma or other malignant tumors is complex; numerous studies have showed that lncRNAs mediated the development of glioma. However, present study cannot state that SNHG16 derived from CSCs is the only mechanism of glioma progress, or CSCs only secrete SNHG16 during glioma progression. At present, exosomes are considered to be an important carrier for lncRNAs, miRNAs, and mRNAs. The present study only showed that exosomal SNHG16 derived from CSCs mediates the development of glioma, however, we cannot state whether CSC secretes SNHG16 through other carriers.

## Conclusion

In conclusion, our study revealed CSC-derived exo-SNHG16 promoted cancer progression by activating the TLR7/MyD88/NFκB/c-Myc signaling pathway, which might be an attractive target in glioma clinical treatment.

## Supplementary Information

**Additional file 1: Supplementary figure 1.** SHG44 and U251 cells were incubated with exosomes isolated from CSCs and CSCs transfected with SNHG16/ si-SNHG16/ NC. (A) qRT-PCR analyzed the expression of SNHG16 in isolated exosomes. (B) The expression of SNHG16 in SHG44 and U251cells was determined. n = 6, *p < 0.05.

## Data Availability

The datasets used and analyzed during the current study are available from the corresponding author on reasonable request.
